# MiR-483 Promotes Colorectal Cancer Cell Biological Progression by Directly Targeting NDRG2 through Regulation of the PI3K/AKT Signaling Pathway and Epithelial-to-Mesenchymal Transition

**DOI:** 10.1155/2022/4574027

**Published:** 2022-01-27

**Authors:** Xifeng Sun, Kun Li, Huiling Wang, Yifang Xia, Ping Meng, Xiaogang Leng

**Affiliations:** ^1^Department of Clinical Laboratory, Weifang People's Hospital, Weifang 261041, China; ^2^Department of Anesthesia, Zhangqiu District People's Hospital, Jinan 250200, China; ^3^Department of Infectious Diseases, Zhangqiu District People's Hospital, Jinan 250200, China; ^4^Department of Imaging, Zhangqiu District People's Hospital, Jinan 250200, China; ^5^Department of Burn and Plastic Surgery, Zhangqiu District People's Hospital, Jinan 250200, China; ^6^Department of Anus and Intestine Surgery, Weifang People's Hospital, Weifang 261041, China

## Abstract

**Background:**

Colorectal cancer is the third frequent tumor in the whole world. MiR-483, located at the 11p15.5 locus, acts as an oncogene in multiple tumors. The purpose of this study is to explore the important roles of miR-483 in colorectal cancer.

**Materials and Methods:**

RT-qPCR and western blot were applied to calculate the mRNA levels of miR-483 and genes. The Kaplan–Meier method was conducted to calculate the survival of patients with colorectal cancer. The proliferation and invasive abilities were measured by Methyl Thiazolyl Tetrazolium (MTT) and transwell assays.

**Results:**

MiR-483 was upregulated in colorectal cancer tissues, and the upregulation of miR-483 predicted poor prognosis of colorectal cancer patients. NDRG2 was a target gene of miR-483 in colorectal cancer. Furthermore, miR-483 has been reported to promote colorectal cancer cell proliferation and invasion through targeting NDRG2 by the PI3K/AKT pathway and epithelial-to-mesenchymal transition (EMT). In addition, the overexpression of miR-483 promoted xenograft growth of LOVO cells.

**Conclusion:**

MiR-483 promoted cell proliferation through the NDRG2/PI3K/AKT pathway and invasion-mediated EMT in colorectal cancer. In view of the multiple mechanisms of molecular immunotherapy, it is necessary to further study the relationship between miR-483 and colorectal cancer, so as to find a more direct and effective treatment method to prevent colorectal cancer.

## 1. Introduction

Colorectal cancer (CRC) is a type of gastrointestinal cancer that is the third frequent tumor in the whole world [1, 2]. Despite the increase of treatment modalities, the metastasis remains to be a challenge for the treatment of colorectal cancer [3]. Therefore, it is urgent to investigate the new biomarkers for the early diagnosis and metastasis of colorectal cancer.

MicroRNAs (miRNAs) are noncoding RNAs with a length of 18–25 nucleotides, which repressed gene expression through directly binding to the mRNA 3′-untranslated region (3′-UTR) at the posttranscriptional level [4, 5]. MiRNAs may act as tumor suppressors or oncogenes to regulate the tumor process including growth, differentiation, and metastasis [6, 7]. A previous study has reported several miRNAs played important roles in colorectal cancer, including miR-483 [8]. MiR-483, which has been reported to be located at the 11p15.5 locus, plays important roles in multiple tumors, including breast cancer, nasopharyngeal carcinoma, and anaplastic thyroid cancer [9–11]. Yang et al. have revealed that, in prostate cancer, miR-483 promoted cell proliferation and invasion [12]. Similarly, Tang et al. have illuminated that miR-483 promoted the proliferation, migration, and invasion and inhibited the apoptosis in hepatocellular carcinoma [13]. Even in colorectal cancer, miR-483 was overexpressed and mediated cellular proliferation by directly targeting DLC-1 [14]. Therefore, we conjectured that miR-483 may promote cell proliferation and metastasis through regulating the PI3K/AKT pathway and EMT in colorectal cancer.

N-Myc downstream-regulated gene 2 (NDRG2) belongs to the NDRG family and is a newly identified differentiation-related gene whose promoter has hypermethylation [15, 16]. NDRG2 played a vital role in multiple biological processes including cell growth, metastasis, and apoptosis [17]. Tamura et al. have indicated that loss of NDRG2 enhanced the metastasis potential in oral squamous cell carcinoma [18]. Moreover, Yamamura et al. have revealed that the suppression of NDRG2 was associated with poor prognosis in gastrointestinal cancer [19]. Even in colorectal cancer, Ali Golestan indicated that overexpression of NDRG2 promoted cell proliferation and invasion [20]. Moreover, Claire Agosta has illuminated that miR-483 promoted the migration and invasion through directly binding to NDRG2 in adrenocortical cancer [21]. Thus, we firmly believe that miR-483 may play an important role in carcinogenesis through NDRG2 in colorectal cancer. In this study, we revealed that miR-483 was upregulated in colorectal cancer and the overexpression of miR-483 predicted poor 5-year survival. MiR-483 promoted the proliferation and invasion in colorectal cancer. In addition, miR-483 promoted growth of CRC cell xenograft.

## 2. Materials and Methods

### 2.1. Sample Collection

*Cancer* tissue samples from 47 patients with colorectal cancer were collected from Weifang People's Hospital. Meanwhile, we also collected the 47 control tissues which were obtained from nonnecrotic colon patients. Patients were excluded if they received chemotherapy or radiation therapy before the blood was drawn. All the samples were immediately frozen in liquid nitrogen and stored at −80°C. Informed consent was obtained from all individual participants included in the study. All the specimens of this study were approved by the Ethical Committee of Weifang People's Hospital.

### 2.2. Cell Culture

Two human colorectal cancer cell lines (LOVO and SW480) and a normal colorectal epithelial cell line CCD-18Co were obtained from the American Type Culture Collection (ATCC, Manassas, VA, USA). All the cells were cultured in the RPMI-1640 medium (Hyclone, UT, USA) with 10% fetal bovine serum (FBS), 100 U/ml penicillin, or 100 mg/ml streptomycin at 37°C in humidified air with 5% CO_2_.

### 2.3. Cell Transfection

The miR-483 mimic and the miR-483 inhibitor, as well as their negative control (NC), were synthesized and purchased from GenePharma (Shanghai, China), which were transfected into colorectal cancer cells VOLO to up- or downregulate the expression of miR-483. The transfection was performed using Lipofectamine 2000 Reagent (Invitrogen, Carlsbad, CA) pursuant to the command of the manufacturer.

### 2.4. RNA Extraction and Real-Time Quantitative Polymerase Chain Reaction (RT-qPCR)

For the miRNAs, total miRNAs were extracted utilizing the miRNeasy Mini Kit (Qiagen, Hilden, Germany) from tissues or cell lines. The reverse transcription was carried out to synthesize the first cDNA chain using the TaqMan miRNA Reverse Transcription Kit (Applied Biosystems, Foster City, CA, USA). Then, the qPCR was performed using the miRNA-specific TaqMan miRNA Assay Kit (Applied Biosystems) on an ABI7500 real-time PCR system (Applied Biosystems). The relative levels of miRNA were derived using the 2^−ΔΔCt^ method with U6 small nuclear RNA as normalization.

For the mRNAs, the TRIzol reagent (Invitrogen) was applied to extract total RNA. The Omniscript Reverse Transcription Kit (Qiagen) was utilized to synthesize the first cDNA chain from total RNAs. The qPCR was carried out using the QuantiTect SYBR Green PCR Kit (Qiagen) on a Quantitect SYBR green PCR system (Qiagen). A method was used for the mRNA quantification, which was normalized by GAPDH. We analyzed the data using the 2^−ΔΔCt^ method for relative quantification. The sequences of primers were as follows: miR-483 forward 5′-AGTTGGCTCACGGTTCTTTCAA-3′, reverse 5′-ATCGCCATGGCCCGCATGTCGG-3′; U6 forward 5′-GCTTCGGCAGCACATATACTAAAAT-3′, reverse 5′-CGCTTCAGAATTTGCGTGTCAT-3′; NDRG2 forward 5′-CCTCACCTC TTCCATTCC-3′, reverse 5′-TATCACCTC CACGCTCAA-3′; and GAPDH, forward 5′-CGGAGTCAACGGATTTGGTCGTAT-3′, reverse 5′-AGCCTTCTCCATGGTGGTGAAGAC-3′.

### 2.5. Western Blotting

Total proteins were extracted using the RIPA buffer (Beyotime, Nantong, China), and then, we tested the protein concentration by bicinchoninic acid protein assay (BCA). Equal amounts of proteins were isolated by 10% sodium dodecyl sulfate polyacrylamide gel electrophoresis (SDS-PAGE) and transferred onto a polyvinylidene fluoride (PVDF) membrane (Millipore, Boston, MA, USA). After blocking with 5% nonfat dried milk for 1h, the membrane was incubated with the primary antibody against NDRG2 (1 : 1000; ab174850, Abcam, Cambridge, USA), E-cadherin (1 : 1000; ab197751, Abcam), N-cadherin (1 : 1000; ab256744, Abcam), vimentin (1 : 1000; ab92547, Abcam), p-PI3K (1 : 1000, 17366, Cell Signaling, San Jose, CA, USA), PI3K (1 : 1000, 3821, Cell Signaling), p-AKT (1 : 1000, 5197, Cell Signaling), AKT (1 : 1000, 4685, Cell Signaling), and GAPDH (1 : 3000, Cell Signaling) at 4°C overnight. Subsequently, the membranes were incubated with the secondary HRP-conjugated antibody (Beyotime) for 2 h at room temperature. Finally, the protein signal was determined with the enhanced chemiluminescence (ECL) kit (Pharmacia Biotech, Arlington, USA).

### 2.6. CCK-8 Assay

The ability of cell proliferation was measured by CCK-8 assay. In brief, 300 *μ*l cell suspension with a concentration of 80% was seeded in each well of the 96-well plates. Meanwhile, CCK-8 reagent (Dojindo, Kumamoto, Japan) was added after 24 h, 48 h, 72 h, or 96 h of culture, and the absorbance at a wavelength of 450 nm was evaluated using a Model 680 Microplate Reader (Bio-Rad, Hercules, CA).

### 2.7. Transwell Assay

Transwell insert (8 *μ*m pore filters, BD Bioscience, Bedford, MA) with a Matrigel (BD Biosciences)-coated membrane was used to calculate the invasion and migration assay. Cells suspended in serum-free media were seeded to the upper chamber, while a normal RPMI-1640 medium with 15% FBS was added in the lower chamber. After incubating for about 24 h at 37°C, the invasive cells were fixed and stained by 4% paraformaldehyde and 10% crystal violet, respectively. Finally, we photographed and counted the invasive cells in five random fields under a microscope (Tokyo, Japan).

### 2.8. Dual-Luciferase Reporter Assay

NDRG2 was predicted to be a potential downstream target of miR-483 using TargetScan (https://www.targetscan.org). The binding sequences were mutated from 5′-AGGGCAGA-3′ to 5′-AGGCGUCA-3′ to validate whether miR-483 directly binds to NDRG2 in colorectal cancer cells. Subsequently, the wild type and the mutant 3′-UTR of NDRG2 were inserted into the dual-luciferase reporter vectors, which were designated as WT or MUT. For the luciferase assay, Lipofectamine 3000 Reagent (Invitrogen, USA) was employed to be cotransfected with the miR-483 mimic and the WT or MUT plasmid into VOLO cells. Then, the luciferase activity was measured on a dual-luciferase reporter assay system (Promega, USA).

### 2.9. Xenograft Tumor Formation Assay

Four-week old nude mice were purchased from Charles River Laboratories (Beijing, China). VOLO cells (5 × 10^6^ cells) were subcutaneously injected into one side of the axillae of the nude mice. The length and the width of the xenograft tumor were evaluated and recorded every 3 days after completing the transplant tumor model. The volume of the xenografts was calculated as the square of length multiplied by the width divided by two. The experiment was terminated after culturing for 26 days, and the xenografts were incised. All animal experiments were performed in the animal laboratory center of Weifang People's Hospital and approved by the Animal Care and Use Committee of Weifang People's Hospital.

### 2.10. Statistical Analysis

All data are expressed as the means ± standard deviation (SD) of at least three independent experiments. Statistical analysis was performed using SPSS 16.0 software (IBM, Armonk, NY, USA). The differences between two or more groups were compared using Student's *t*-test or one-way ANOVA. The association between the expression of miR-483 and the overall survival for colorectal cancer patients were assessed by the Kaplan–Meier curve and log-rank test. Results were considered statistically significant if *P* < 0.05. Each experiment was repeated three times.

## 3. Results

### 3.1. Upregulation of MiR-483 Predicted Poor Prognosis of Colorectal Cancer

The mRNA level of miR-483 was calculated in 47 pairs of colorectal cancer and nonnecrotic colon tissues. As expected, the expression of miR-483 was higher in colorectal cancer tissues in comparison with corresponding nonnecrotic colon tissues (*P* < 0.05) (Figure 1(a)). In addition, the overexpression of miR-483 predicted poor 5-year survival in colorectal cancer (*P* < 0.05) (Figure 1(b)).

### 3.2. MiR-483 Promoted the Proliferation and Invasion in Colorectal Cancer Cells

The expression of miR-483 was assessed in two colorectal cancer cell lines (LOVO and SW480) and a normal colorectal epithelial cell line CCD-18Co. Similar with the findings in tissues, miR-483 was overexpressed in CCD-18Co cells compared with colorectal cancer cell lines LOVO (*P* < 0.05) and SW480 (*P* < 0.05) (Figure 2(a)). To explore the functions of miR-483 in colorectal cancer, the miR-483 mimic or the miR-483 inhibitor was transfected in LOVO cells to up- (*P* < 0.01) or downregulate (*P* < 0.05) miR-483 (Figure 2(b)).

MTT assay revealed that the miR-483 mimic promoted cell proliferation (*P* < 0.05), while the cell proliferative ability was suppressed by the miR-483 inhibitor in LOVO cells (*P* < 0.05) (Figure 2(c)). Furthermore, transwell assay illuminated that the miR-483 mimic enhanced the cell invasive ability (*P* < 0.01) while the miR-483 inhibitor suppressed (*P* < 0.05) (Figure 2(d)). All the findings elucidated that miR-483 promoted the capacities of proliferation and invasion in colorectal cancer cell line LOVO.

### 3.3. MiR-483 Regulated the Expression of NDRG2 through Directly Binding to the 3′-UTR of NDRG2 mRNA

TargetScan predicted NDRG2 was a target gene of miR-483 and the binding site was located at 3′-UTR of NDRG2 mRNA. To validate miR-483 direct binding to the potential binding site of NDRG2, the binding sequences were mutated from 5′-AGGGCAGA-3′ to 5′-AGGCGUCA-3′ and then inserted into the luciferase vectors (Figure 3(a)). The luciferase reporter assay indicated that the luciferase activity of LOVO cells transfected with the wild-type NDRG2 3′-UTR was decreased by miR-483 mimic (*P* < 0.05), while the miR-483 mimic has no effect on the luciferase activity of cells transfected with mutant NDRG2 3′-UTR (*P* < 0.05) (Figure 3(b)). Furthermore, the mRNA levels of NDRG2 were measured when transfected with the miR-483 mimic or the miR-483 inhibitor in LOVO cells. As expected, the overexpression of miR-483 enhanced the mRNA level of NDRG2 (*P* < 0.05), while the knockdown of miR-483 inhibited the expression of NDRG2 in LOVO cells (*P* < 0.05) (Figure 3(c)). All the results illuminated that miR-483 regulated the expression of NDRG2 in colorectal cancer cell line LOVO.

### 3.4. MiR-483 Promoted the EMT and Activated the Phosphorylation of the PI3K/AKT Signaling Pathway

The relative mRNA level of NDRG2 was calculated, and it was found to be upregulated in nonnecrotic colon tissues in comparison with that of colorectal cancer tissues (*P* < 0.05) (Figure 4(a)). Also, the expression of NDRG2 was detected in normal colorectal epithelial cell line CCD-18Co and two human colorectal cancer cell lines LOVO and SW480. Not unfortunately, the expression of NDRG2 was lower in LOVO (*P* < 0.05) and SW480 (*P* < 0.05) cells than that in CCD-18Co cells (Figure 4(b)). Moreover, western blot was conducted to assess the expressions of EMT and PI3K pathway associated proteins in LOVO cells. We discovered that the miR-483 mimic promoted the EMT via NDRG2 by suppressing the expression of NDRG2 and N-cadherin while improving the expression of E-cadherin in LOVO cells (Figure 4(c)). Phosphorylation of PI3K and AKT promoted cell growth, proliferation, and survival [22]. As we expected, the overexpression of miR-483 enhanced the expression of p-PI3K and p-AKT in LOVO cells (Figure 4(d)), which elucidated that miR-483 activated the phosphorylation of the PI3K/AKT signaling pathway.

### 3.5. MiR-483 Enhanced the Xenograft Growth In Vivo

LOVO cells stably transfected with the miR-483 mimic, or control plasmid was applied to inject into the nude mice subcutaneously. The xenograft tumor volume was calculated every 3 days, and the group of transfecting the miR-483 mimic had a higher growth rate than the control group (Figure 5(a)). After dissecting the nude mice, the xenograft tumors were collected and the volumes were calculated. Also, we discovered the tumor volumes of cells overexpressing miR-483 was bigger than that of the control group, which indicated that miR-483 mimic promoted the growth of colorectal cancer xenograft (*P* < 0.05) (Figure 5(b)).

## 4. Discussion

Colorectal cancer is the third frequent tumor and one of the leading causes of cancer-related death worldwide [1, 2]. The morbidity and mortality of colorectal cancer caused by metastasis are increasing rapidly [3, 23]. Therefore, it is urgent to explore the early diagnosis and metastasis of newly biomarkers for colorectal cancer.

MiRNAs repressed the protein degradation and translation through directly binding to the 3′-UTR of target mRNA at the posttranscriptional level [24]. MiR-483 which acted as a prognostic biomarker was upregulated in esophageal squamous cell carcinoma [25]. Consistent with the findings, we discovered that miR-483 was upregulated in colorectal cancer tissues in comparison with the nonnecrotic colon tissues. Moreover, miR-483 may act as a prognosis marker and the overexpression of miR-483 predicted a poor 5-year overall survival of colorectal cancer patients, which was the first time to propose the association between miR-483 and the survival of CRC. Furthermore, miR-483 played an oncogenic role and promoted cell proliferation and migration in esophageal squamous cell carcinoma [26]. In adenocarcinoma, Song et al. indicated that miR-483 promoted cell invasion and the EMT [27]. Our results were consistent with all the findings that the overexpression of miR-483 in colorectal cancer promoted cell proliferation and invasion, while the reverse was downregulation. However, miR-483 served a tumor suppressive role in glioma [28], and we speculated that miR-483 has a tissue-specific expression. In addition, we first proposed that miR-483 promoted the growth of colorectal cancer cell xenografts.

NDRG2 is a gene with promoter hypermethylation and is a newly identified differentiation-related gene [15, 16]. In esophageal cancer, NDRG2 inhibited cell proliferation, migration, invasion, and the EMT [17]. NDRG2 was a target gene of several miRNAs including miR-141b, miR-375, miR-301, and miR-650 [29–32]. Consistent with the findings of Claire Agosta in adrenocortical cancer [21], we discovered that NDRG2 was a target gene of miR-483 and miR-483 mediated the expression of NDRG2 in colorectal cancer. The expression of NDRG2 was lower in colorectal cancer tissues than in nonnecrotic colon tissues. Moreover, miR-483 promoted colorectal cancer cell proliferation, invasion, and EMT through targeting NDRG2 and activated the PI3K/AKT pathway.

## 5. Conclusions

MiR-483 promoted colorectal cancer cell proliferation, invasion, and EMT through directly targeting NDRG2 and activated the PI3K/AKT pathway. In addition, the overexpression of miR-483 promoted the growth of LOVO cells xenograft. Our data suggest that miR-483 is a prognostic predictor and can serve as a potential therapeutic target of colorectal cancer.

## Figures and Tables

**Figure 1:** Upregulation of miR-483 predicted poor prognosis of colorectal cancer. (a) The expression of miR-483 was higher in colorectal cancer tissues than in the nonnecrotic colon tissues. (b) Overexpression of miR-483 predicted poor 5-year survival of colorectal cancer patients. ^*∗*^*P* < 0.05. NT: normal tissues; CRC: colorectal cancer.

**Figure 2:** MiR-483 promoted the proliferation and invasion in colorectal cancer cells. (a) MiR-483 was overexpressed in CCD-18Co cells versus LOVO and SW480 cells. (b) The miR-483 mimic or the miR-483 inhibitor was transfected to up- or downregulate miR-483 in LOVO cells. (c) MTT assay revealed that the miR-483 mimic promoted the proliferation in LOVO cells. (d) The invasive ability was enhanced by the miR-483 mimic cell, while it was inhibited by the miR-483 inhibitor in LOVO cells. ^*∗*^*P* < 0.05; ^*∗∗*^*P* < 0.01.

**Figure 3:** MiR-483 regulated the expression of NDRG2 through binding to NDRG2 mRNA 3′-UTR. (a) TargetScan predicted NDRG2 was a target gene of miR-483 and the binding site was located at the 3′-UTR of NDRG2 mRNA. (b) The luciferase reporter assay indicated that miR-483 directly targeted NDRG2 in LOVO cells. (c) Overexpression of miR-483 enhanced the mRNA level of NDRG2, while the knockdown of miR-483 inhibited the expression of NDRG2 in LOVO cells. ^*∗*^*P* < 0.05; ^#^*P* < 0.05.WT: wild type; MUT: mutant type.

**Figure 4:** MiR-483 promoted the EMT and activated the phosphorylation of the PI3K/AKT signaling pathway. (a) The mRNA level of NDRG2 in nonnecrotic colon tissues was higher than that in colorectal cancer tissues. (b) NDRG2 was lowly expressed in colorectal cancer cells than normal cells. (c) Western blot illuminated that miR-483 promoted the EMT through NDRG2. (d) MiR-483 activated the PI3K/AKT pathway. ^*∗*^*P* < 0.05. NT: normal tissues; CRC: colorectal cancer; N-Ca : N-cadherin; E-Ca : E-cadherin; and GAPDH: glyceraldehyde-phosphate dehydrogenase.

**Figure 5:** MiR-483 enhanced the growth of xenograft in vivo. (a) MiR-483 promoted colorectal cancer growth in vivo. (b) The tumor volume of cells overexpressing miR-483 was bigger than the control group. ^*∗*^*P* < 0.05.

## Data Availability

Data supporting the findings of this study are available on reasonable request from the corresponding author.
